This article has been retracted.

# Molecular Mechanism of 73HOXC-AS1-Activated Wnt*β*-Catenin Signaling and eIF4AIII in Promoting Progression of Gastric Cancer

**DOI:** 10.1155/2021/8814843

**Published:** 2021-04-15

**Authors:** Shumin Zhang, Lianzhen Wang, Yuting Gao, Yanxia Fan, Gang Zhang, Yujie Zhang

**Affiliations:** ^1^Department of Gastroenterology, The Fourth People's Hospital of Jinan, Jinan 250031, China; ^2^Gastrointestinal Surgery, The Fourth People's Hospital of Jinan, Jinan 250031, China; ^3^Department of Nursing, The Fourth People's Hospital of Jinan, Jinan 250031, China; ^4^Department of Neurology, The Fourth People's Hospital of Jinan, Jinan 250031, China; ^5^Department of General Surgery, The Fourth People's Hospital of Jinan, Jinan 250031, China

## Abstract

**Objective:**

This study is aimed at exploring the regulatory mechanism of 73HOXC-AS1 overexpression plasmid-activated Wnt*β*-catenin classic signaling pathway and eukaryotic initiation factor 4A (eIF4AIII) expression increased by lentivirus-eIF4AIII-RNAi (44682-1) (LV-eIF4AIII-RNAi (44682-1)).

**Methods:**

Focusing on the occurrence and progression of gastric cancer, the human gastric cancer cell line BGC823 (University Experimental Center) was taken as the research object and was transfected after subculture. According to the different ways of transfection, the cells were divided into the P1 group (LV-eIF4AIII-RNAi (44682-1) overexpressed plasmid), the P2 group (pcDNA-HOXC-AS1 overexpressed plasmid), the P3 group (LV-eIF4AIII-RNAi (44682-1) + pcDNA-HOXC-AS1), and the P4 group (no transfection, control group). Cell proliferation was detected by CCK-8 (Cell Counting Kit-8) assay, Western blotting was adopted to detect Wnt3a and P-GSK3*β* proteins, Transwell assay was adopted to detect the ability of cell migration and invasion, and cell cycle and apoptosis were detected by flow cytometry.

**Results:**

The results show that the protein expression levels of Wnt3a and P-GSK3*β* (glycogen synthase kinase-3*β*) in the P1 and P4 groups were lower than those in the P2 and P3 groups (*P* < 0.05). The cell activity and clone number of BGC823 in the P3 group were higher than those in the P1, P2, and P4 groups (*P* < 0.05). The apoptosis rate of BGC823 cells in the P3 group was significantly higher than those in the P1, P2, and P4 groups (*P* < 0.05). The proportion of BGC823 cells in the P3 group at the S phase was significantly higher than those in the P1, P2, and P4 groups, while the proportion in the G2 phase was significantly lower than those in the P1, P2, and P4 groups (*P* < 0.05). The number of migrating and invading BGC823 cells in the P3 group was significantly higher than those in the P1, P2, and P4 groups, while the number of migrating BGC823 cells in the P4 group was significantly lower than those in the P1 and P2 groups (*P* < 0.05).

**Conclusion:**

The 73HOXC-AS1 overexpression plasmid-activated Wnt*β*-catenin classic signaling pathway and eIF4AIII expression increased by LV-eIF4AIII-RNAi (44682-1) could act together on BGC823 cells to improve cell proliferation activity, migration, and invasion; inhibit cell apoptosis; and prevent cells from entering the S phase.

## 1. Introduction

Gastric cancer is a malignant tumor originating from the epithelium of the gastric mucosa, and its incidence ranks first among all kinds of tumors in my country. More than 70% of early gastric cancer has no obvious symptoms, and with the progression of the disease, nonspecific symptoms similar to gastritis or gastric ulcer may gradually appear, including upper abdominal discomfort or dull pain, pantothenic acid, belching, nausea, occasionally vomiting, loss of appetite, indigestion, and melena [1–3]. The pathological type of gastric cancer is mainly adenocarcinoma, followed by squamous cell carcinoma, adenosquamous carcinoma, carcinoid, and small-cell carcinoma. The current cause of the disease is still unclear, and it may be related to a variety of factors, such as lifestyle, diet, environmental factors, genetic quality, and spiritual factors. It is also related to chronic gastritis, gastric polyps, gastric mucosal dysplasia, intestinal metaplasia, and postoperative remnant stomach [4]. Metastasis is the most essential manifestation of gastric cancer. Once the cancer invades the serous membrane, it will invade neighboring organs or tissues such as the liver, pancreas, spleen, transverse colon, jejunum, diaphragm, greater omentum, and abdominal wall [5]. Cancer cells can also be planted in the abdominal cavity, pelvic cavity, ovary, and rectal bladder lacuna when they fall off. Clinical data shows that about 90% of gastric cancer patients die because of tumor metastasis [6, 7]. Therefore, in order to improve the high mortality rate of cancer, knowing how to prevent and control gastric cancer tumors is extremely important. Glycogen synthase kinase-3 (GSK-3) is an evolutionarily conserved serine/threonine kinase that is ubiquitous in mammalian eukaryotic cells. In addition to regulating the activity of glycogen synthase (GS), GSK-3*β* also acts on a number of signaling proteins, structural proteins, and transcription factors, regulating cell differentiation, proliferation, survival, and apoptosis. In the research of many major diseases such as neurodegenerative diseases of cancer and neuropsychiatric diseases, more and more researchers pay attention to it as a therapeutic target. The positive expression rates of Wnt2b, *β*-catenin, and cyclin D1 in gastric cancer tissues were significantly higher than those in normal gastric tissues and adjacent tissues.

The transcription factors encoded by Hox play an important role in the carcinogenesis of normal tissues. Previous cDNA microarray detection results showed that HoxC6 expression was significantly upregulated in gastric cancer tissues compared with adjacent tissues. The expression level of HoxC6 mRNA in gastric cancer tissues decreased, and its expression was closely related to lymph node metastasis. The expression level of EIF4A1 in gastric cancer tissues with lymph node metastasis was higher than that in adjacent normal tissues. Silvestrol did not affect proliferation and survival of SGC-7901 cells but inhibited cell invasion and migration. The mechanism may be related to silvestrol's regulation of the AKT signaling pathway.

Long noncoding RNAs (lncRNA) refer to a class of transcripts with a size of 200 nucleotides that have no coding protein function, which can control gene expression in many aspects such as heredity and transcription level. In malignant tumors, it can be used as a carcinogen or tumor suppressor to participate in gene transcription, vascular invasion, and other processes [8, 9]. Among them, HOXC-AS1 is the earliest discovered lncRNA closely related to tumor metastasis and poor prognosis, and it may also play an important biological role in the progression of gastric cancer [10]. The Wnt protein family is a widespread secreted glycoprotein with 19 members, which play a huge role in animal growth and cell proliferation and differentiation. Wnt3a participates in the Wnt*β*-catenin classic signaling pathway, and it regulates the occurrence and progression of tumors [11, 12]. At present, the inhibition of the Wnt*β*-catenin classic signaling pathway is also a hotspot in antitumor research. The eukaryotic translation initiation factor eIF4A is a protein that binds to the small ribosomal subunit at the translation initiation phase and contains two RecA-like domains and an intermediate hinge region [13]. Studies have found that changes in eIF4AIII gene levels can throw protein translation out of control, which in turn causes the occurrence and progression of cancer. Therefore, it is inferred that eIF4AIII may become a potential target of anticancer therapy [14]. Based on that, the 73HOXC-AS1 was adopted to activate the Wnt*β*-catenin pathway and silence the eIF4AIII gene to comprehensively analyze the molecular mechanism of gastric cancer progression. In this study, the human gastric cancer cell line BGC823 from the Experimental Center of our university was selected as the research object, and it was cultured and subcultured in Dulbecco's modified Eagle's (DMEM) medium containing 10% fetal bovine serum at 37°C and 5% carbon dioxide. According to different ways of transfection, the cultured cells are divided into the P1 group, the P2 group, the P3 group, and the P4 group. By comparing the proliferation activity, apoptosis rate, cell cycle ratio, migration and invasion ability of different groups of cells, and Wnt3a and P-GSK3*β* protein levels, the molecular mechanism of the 73HOXC-AS1 overexpression plasmid-activated Wnt*β*-catenin classic signaling pathway and LV-eIF4AIII-RNAi (44682-1)-increased eIF4AIII expression on gastric cancer BGC823 cells was comprehensively evaluated.

In summary, the prevention and treatment of gastric cancer are still a topic of concern at present, and a discussion at the molecular level will help to better understand the occurrence and progression of gastric cancer.

## 2. Materials and Methods

### 2.1. Cell Source and Grouping

The human gastric cancer cell line BGC823 from the Experimental Center of our university was selected as the research object, and it was cultured and subcultured in DMEM medium containing 10% fetal bovine serum at 37°C and 5% carbon dioxide. According to the different ways of transfection, the cells were divided into the P1 group (LV-eIF4AIII-RNAi (44682-1) overexpressed plasmid), the P2 group (pcDNA-HOXC-AS1 overexpressed plasmid), the P3 group (LV-eIF4AIII-RNAi (44682-1) + pcDNA-HOXC-AS1), and the P4 group (no transfection, control group).

### 2.2. Cell Transfection

We have the P1 group (LV-eIF4AIII-RNAi (44682-1) overexpression plasmid), the P2 group (pcDNA-HOXC-AS1 overexpression plasmid), the P3 group (LV-eIF4AIII-RNAi (44682-1) + pcDNA-HOXC-AS1), and the P4 group (untransfected, control group). The Cell Counting Kit-8 (CCK-8) method was adopted to detect cell proliferation. Cells were transfected when 90% of them were grown in 75 cm^2^ flasks. First, four wells with good cell fusion were selected from a 6-well plate, and the wells were marked and grouped. According to the calculated amount, 100 *μ*L of 1 : 200 diluted polybrene gene transfection enhancer was added. Then, the corresponding lentivirus particle mixture (LV-eIF4AIII-RNAi (44682-1)) and pcDNA-HOXC-AS1 overexpressed plasmid were added, respectively. The blank control group was added with 1 mL antibiotic-free BGC823 cell culture medium and cultured at 37°C and 5% carbon dioxide for 12 hours. After that, the medium in the orifice plate was removed with a 1000 *μ*L pipette, and then washed with 1 mL phosphate buffer. Five mL of BGC823 cell culture medium containing antibiotics and 10% fetal bovine serum was added. When the cell fusion was over 80%, the cell suspension was prepared and transfected successfully.

The transfection steps were as follows:

- Cell culture: 6 cm cell dishes were taken, and 2 mL culture medium containing 1 ~ 2 × 10^5^ cells was added into each well. The culture density would be up to 40%~60% cultured with CO_2_ at 37°C. If the density was too high, it was unfavorable to select cells after transfection
- Transfer dye preparation: the following two liquids (the amount used for transfection of each well cell) were configured in an EP tube. Liquid A: 1 *μ*g plasmid DNA was diluted with serum-free medium. Liquid B: 2 *μ*L liposomes was diluted with serum-free medium. Liquids A and B were gently mixed and left for 5 minutes
- Liquid B was added to liquid A, mixed with light elastic, and left at room temperature for 10-15 minutes
- Preparation for transfection: cells were rinsed twice with 1 mL serum-free medium, then added with 4 mL serum-free medium
- Transfection: the A/B complex was slowly added to the culture medium, shaken well, and placed in a 37°C incubator for 6~24 hours. The serum-free solution was absorbed and transferred to the normal culture medium for further culture
- After transient transfection, cell proteins or RNA could be extracted after the cells were overgrown for 48 h-72 h to verify the knockdown/overexpression efficiency

### 2.3. Detection of Protein Levels of Wnt3a and P-GSK3*β*

Western blotting was used to detect the protein levels of Wnt3a and P-GSK3*β*. When the cells grow to 90%, the centrifuge tube could be collected and centrifuged at 1200 r/min for 5 minutes, and the supernatant was then discarded. 300 *μ*L radio immunoprecipitation assay lysate containing protease inhibitors was added, and then crushed into polypropylene tubes. The supernatant was obtained by centrifugation at 1200 r/min for five minutes, which was the protein extract. Then, a group of bovine serum protein solutions with concentrations of 0.10 mg/mL, 0.08 mg/mL, 0.06 mg/mL, 0.04 mg/mL, 0.02 mg/mL, and 0 mg/mL were prepared. The absorbance of this group of solutions was measured, and a standard curve of protein concentration to absorbance was obtained. The protein concentration was obtained according to the standard curve.

### 2.4. BGC823 Cell Proliferation Detection

Cell proliferation was measured by CCK-8. The cultured cells were digested and centrifuged, and 5 mL BGC823 cell culture medium containing antibiotics and 10% fetal bovine serum was then added to each group of cells. A 10 *μ*L cell suspension was absorbed into a 10 *μ*L dye tube, mixed well, and dropped onto the cell counting board for flow cytometry counting. The cell concentration was adjusted to 4 × 10^4^ cells/mL, 100 *μ*L of which was inoculated in a 96-well plate, 10 *μ*L CCK-8 solution was added to culture for 1 hour, and the absorbance value (OD) of each well was determined at the wavelength of 450 nm. The transfected cells were inoculated in 6-well plates at a density of 600 cells/well 24 hours after transfection, and cultured for 3 weeks. Fixed with pure methanol for 20 minutes, the cells were stained with 0.1% crystal violet for 20 minutes, dried, photographed, and the number of clones counted.

### 2.5. BGC823 Cell Cycle Distribution and Apoptosis Detection

The cells were added with 3 mL 0.3% trypsin digestion solution and placed in an incubator with 5% carbon dioxide at 37°C for 10 minutes. The cells were neutralized in double volume BGC823 cell culture medium, fixed with alcohol, and centrifuged at 1200 r/min for 5 minutes. A 1000 *μ*L pipette was added to filter the cells into the flow tube through a 200-mesh nylon mesh, and 10 *μ*L RNase endonuclease was added to each tube. The cells were then immersed in a water bath at 37°C for half an hour. Then, 400 *μ*L propidium iodide staining solution was added, and cell cycle distribution (S, G1, and G2 phase) was detected by flow cytometry half an hour later.

#### 2.5.1. Apoptosis Experiment

The cells in each group were blown evenly with 5 mL phosphate buffer, and the concentration was adjusted to 5 × 10^6^ cells/mL. A filtering through a 200-mesh nylon mesh into a 1000 *μ*L flow pipe, the cells were centrifuged at 1200 r/min for 5 minutes to discard the supernatant. 100 *μ*L binding buffer suspension cells and 5 *μ*L Annexin V labeled with red fluorescent dye phycoerythrin were added into each tube. After they were washed well, they were left to react for 20 minutes at room temperature and detection was accomplished by flow cytometry automatically.

### 2.6. Transwell Chamber Assay for Detecting Cell Migration and Invasion Ability

#### 2.6.1. Migration Experiment

The logarithmic growth phase cells were prepared into a 5 × 10^5^/mL cell suspension, and a 500 *μ*L DMEM medium was added to the Transwell chamber. A 200 *μ*L cell suspension was added to the upper chamber and fixed with paraformaldehyde for half an hour after 24 h of culture. 0.1% methyl violet staining was conducted for half an hour, and the water droplets on the surface of the film was dried. Eight high-definition fields of view were counted under the microscope, and the average value was calculated. In the invasion experiment, 2.5% matrix glue was prepared at 4°C using antibiotic-and-serum-free BGC823 cell culture medium. 100 *μ*L matrix glue was laid in each Transwell chamber and 100 *μ*L type V collagen was added. Then, the samples were cultured at 37°C for 1 hour, and the counting method was the same as that in the migration experiment after drying.

### 2.7. Statistical Methods

The data processing in this study was analyzed by SPSS version 19.0 statistical software, the measurement data was expressed as mean plus or minus standard deviation $\left(\bar{x}\pm s\right)$, and the counting data was expressed as percentage (%). The proliferation activity, apoptosis rate, cycle ratio (the S, G1, and G2 phases), and migration and invasion ability of cells in the P1, P2, P3, and P4 groups, as well as Wnt3a and P-GSK3*β* protein levels were compared by analysis of variance. *P* < 0.05 indicated statistical significance, and Origin 8.0 was adopted for mapping.

## 3. Results

### 3.1. Protein Expression Levels of Wnt3a and P-GSK3*β* in Cells

The protein expression levels of Wnt3a and P-GSK3*β* in the P1 and P4 groups were significantly lower than those in the P2 and P3 groups (Figure 1), and the differences were statistically significant (*P* < 0.05). There was no statistically significant difference in Wnt3a and P-GSK3*β* protein expression between the P2 and P3 groups (*P* > 0.05), or between the P1 and P4 groups (*P* > 0.05). The protein expression of P1 was evidently lower than that of P3 or P4, with statistical significance (*P* < 0.05).  Figure 2 shows the Wnt3a and P-GSK3*β* protein bands in cells, and those in the P1 and P4 groups are significantly brighter than those in the P2 and P3 groups. The brightness of the Wnt3a and P-GSK3*β* bands in the P2 and P3 groups was similar.

### 3.2. Cell Viability and Clone Number Results

Only after 10 h, there was a notable difference in the proliferative activity of each group.  Figure 3 shows that the BGC823 cell activity and clone number were significantly higher in the P3 group than in all the other groups, and the difference was notably significant (*P* < 0.05). The cell activity and clone number of BGC823 in the P4 group were significantly lower than those in P1 and P2 groups, with statistically significant difference (*P* < 0.05). There was no significant difference in BGC823 cell activity and clone number between the P1 and P2 groups (*P* > 0.05).

### 3.3. BGC823 Cell Cycle

Figure 4 illustrates that the proportion of BGC823 cells in the S phase is significantly higher in the P3 group than in all the other groups, and the difference is statistically significant (*P* < 0.05). The proportion of BGC823 cells in the S phase is significantly lower in the P4 group than in the P1 and P2 groups, with statistically significant difference (*P* < 0.05). There was no significant difference in the proportion of BGC823 cells in the G1 phase among all groups (*P* > 0.05). The proportion of BGC823 cells in the G2 phase is significantly lower in the P3 group than in all the other groups, with a statistically significant difference (*P* < 0.05). The proportion of BGC823 cells in the G2 phase was significantly higher in the P4 group than in the P1 and P2 groups, with a statistically significant difference (*P* < 0.05). The proportion of BGC823 cells in the S, G1, and G2 phases in the P1 and P2 groups is not statistically significant (*P* > 0.05).

### 3.4. Comparison of BGC823 Cell Apoptosis

Figure 5 shows that the apoptosis rate of BGC823 cells in the P3 group is the highest among all groups, and the difference is statistically notable (*P* < 0.05). The apoptosis rate of BGC823 cells in the P4 group was significantly lower in contrast to the P1 and P2 groups, with statistically significant difference (*P* < 0.05). The apoptosis rate of BGC823 cells in the P1 and P2 groups was not statistically notable (*P* > 0.05).

### 3.5. Comparison of BGC823 Cell Migration

Figure 6 shows that the number of BGC823 cells migrating in the P3 group is the highest among all groups, and the difference is statistically significant (*P* < 0.05). The number of BGC823 cells migrating in the P4 group was obviously lower than that in the P1 and P2 groups, and the difference was statistically significant (*P* < 0.05). There was no statistically significant difference in the number of BGC823 cells migrating between the P1 and P2 groups (*P* > 0.05).  Figure 7 shows the cell migration images of the four groups. The P3 group had the most number of migrating cells, which was significantly more compared to the other groups, while the P4 group had the least number of migrating cells.

### 3.6. Comparison of BGC823 Cell Invasion

Figure 8 shows that the number of invading BGC823 cells in the P3 group is the highest among all groups, and the difference is statistically significant (*P* < 0.05). The number of invading BGC823 cells was obviously lower in the P4 group than in the P1 and P2 groups, and the difference was statistically significant (*P* < 0.05). There was no statistically significant difference in the number of invading BGC823 cells between the P1 and P2 groups (*P* > 0.05).  Figure 9 shows the images of cell invasion of the four groups. The P3 group had the most number of invading cells, which was remarkably higher compared to the other groups, while the P4 group had the least number of invading cells, which corresponded to the above quantitative data results.

## 4. Discussion

Gastric cancer, as one of the common malignant tumors of the digestive tract, poses great harm to people's life and health. However, as the occurrence and progression of gastric cancer are the biological results of multiple factors, the traditional single treatment has always been unable to play a satisfactory therapeutic effect. Therefore, it is necessary to conduct an in-depth study on gastric cancer gene molecules [15, 16]. In this study, the human gastric cancer cell BGC823 was transfected with LV-eIF4AIII-RNAi (44682-1) and pcDNA-HOXC-AS1 overexpressed plasmids. It was found that the expression levels of Wnt3a and P-GSK3*β* in the P1 and P4 groups were significantly lower than those in the P2 and P3 groups (*P* < 0.05), and the differences in Wnt3a and P-GSK3*β* protein expression levels in the P2 and P3 groups were not statistically significant (*P* > 0.05), which was different from the research results of Dong et al. in 2019 [17]. Wnt3a and P-GSK3*β* are the major proteins involved in activating Wnt*β*-catenin classical signaling pathways, and cells transfected with 73HOXC-AS1 overexpressed plasmid could enhance the expression of Wnt3a and P-GSK3*β* proteins, thereby activating the Wnt*β*-catenin signaling pathway [18]. The cell activity and clone number of BGC823 were significantly higher in the P3 group than in the P1, P2, and P4 groups (*P* < 0.05), while the differences in cell activity and clone number between the P1 and P2 groups were not statistically significant (*P* > 0.05). This indicated that 73HOXC-AS1 overexpression plasmid-activated Wnt*β*-catenin classic signaling pathway and eIF4AIII expression increased by LV-eIF4AIII-RNAi (44682-1) could act together on BGC823 cells to improve cell proliferation activity [19].

The proportion of BGC823 cells at the S phase was significantly higher in the P3 group than in the P1, P2, and P4 groups, while the proportion at the G2 phase was significantly lower than that in the P1, P2, and P4 groups (*P* < 0.05). It was similar to the research results of Zhu et al. in 2019 [20]. The S phase refers to the DNA replication phase, which mainly involves the replication of genetic material, namely, the synthesis of DNA, histones, and enzymes needed for replication. The increase in the number of cells at the S phase means that the proliferation and differentiation activities of the cells are enhanced. Therefore, the 73HOXC-AS1 overexpression plasmid-activated Wnt*β*-catenin classic signaling pathway and eIF4AIII expression increased by LV-eIF4AIII-RNAi (44682-1) could accelerate the cell proliferation cycle and increase the cell ratio in the S phase [21–23]. The number of migrating BGC823 cells was significantly higher in the P3 group than in the P1, P2, and P4 groups, while the number of migrating cells was significantly lower in the P4 group than in the P1 and P2 groups (*P* < 0.05). This was similar to the research results of Wu et al. in 2019 [24]. The results showed that the 73HOXC-AS1 overexpression plasmid-activated Wnt*β*-catenin classic signaling pathway and eIF4AIII expression increased by LV-eIF4AIII-RNAi (44682-1) could greatly improve the cell migration ability. From the cell migration image, the P3 group had the largest number of migrating cells, which was significantly higher compared to those of the other groups. However, the P4 group had the least number of migrating cells, which corresponded to the quantitative data above. The number of invading BGC823 cells was significantly higher in the P3 group than in the P1, P2, and P4 groups, and the difference was statistically significant (*P* < 0.05). And there was no statistically significant difference in the number of invading BGC823 cells between the P1 and P2 groups (*P* > 0.05). These results suggested that the 73HOXC-AS1 overexpression plasmid-activated Wnt*β*-catenin classic signaling pathway and eIF4AIII expression increased by LV-eIF4AIII-RNAi (44682-1) had similar effects on cancer cells, while the combined adoption of the two would better improve the invasion ability of cells [25].

## 5. Conclusion

In this study, the human gastric cancer cell line BGC823 was subcultured and divided into the P1 group (LV-eIF4AIII-RNAi (44682-1) overexpressed plasmid), the P2 group (pcDNA-HOXC-AS1 overexpressed plasmid), the P3 group (LV-eIF4AIII-RNAi (44682-1) + pcDNA-HOXC-AS1), and the P4 group (no transfection, control group) according to the different ways of transfection. The results showed that the 73HOXC-AS1 overexpression plasmid-activated Wnt*β*-catenin classic signaling pathway and eIF4AIII expression increased by LV-eIF4AIII-RNAi (44682-1) could act together on BGC823 cells to improve the cell proliferation activity, migration, and invasion; inhibit cell apoptosis; and prevent cells from entering the S phase. However, it was only discussed at the cell level and no in vivo experiments were carried out. Therefore, mice were selected as research objects to further analyze the regulatory effect of 73HOXC-AS1 combined with eIF4AIII on gastric cancer. In conclusion, this study provided a theoretical basis for the study of molecular regulatory mechanisms of the occurrence and progression of gastric cancer.

## Figures and Tables

**Figure 1:** Wnt3a and P-GSK3*β* protein expression levels in cells. (Note: (a) is the expression of the Wnt3a protein; (b) is the expression of the P-GSK3*β* protein. ∗ indicates that the difference is statistically significant compared to the P2 group (*P* < 0.05)).

**Figure 2:** Wnt3a and P-GSK3*β* protein bands. (Note: (a) is the Wnt3a protein band; (b) is the P-GSK3*β* protein band).

**Figure 3:** Comparison of cell proliferation activity and clone number of four groups. (Note: (a) is the cell proliferation activity of the four groups; (b) is the number of cell clones in the four groups. ∗ indicates that the difference is statistically significant compared to the P3 group (*P* < 0.05); # indicates that the difference is statistically significant compared to the P4 group (*P* < 0.05)).

**Figure 4:** Cell cycle comparison of four groups of BGC823 cells. (Note: (a) is the proportion of cells in the S phase; (b) is the proportion of cells in the G1 phase; (c) is the proportion of cells in the G2 phase; ∗ indicates that the difference is statistically significant compared to the P3 group (*P* < 0.05); # indicates that the difference is statistically significant compared to the P4 group (*P* < 0.05).

**Figure 5:** Cell cycle comparison of four groups of BGC823 cells. (Note: ∗ indicates that the difference is statistically significant compared to the P3 group (*P* < 0.05); # indicates that the difference is statistically significant compared to the P4 group (*P* < 0.05).

**Figure 6:** Comparison of the migration of the four groups of BGC823 cells. (Note: ∗ indicates that the difference is statistically significant compared to the P3 group (*P* < 0.05); # indicates that the difference is statistically significant compared to the P4 group (*P* < 0.05).

**Figure 7:** Four groups of BGC823 cell migration images (×400).

**Figure 8:** Comparison of the BGC823 cell invasion in four groups. (Note: ∗ indicates that the difference is statistically significant compared to the P3 group (*P* < 0.05); # indicates that the difference is statistically significant compared to the P4 group (*P* < 0.05).

**Figure 9:** Four groups of BGC823 cell migration images (×400).

## Data Availability

Some or all data, models, or code generated or used during the study are available from the corresponding authors on request.
